# Prediction of the Least Principal Stresses Using Drilling Data: A Machine Learning Application

**DOI:** 10.1155/2021/8865827

**Published:** 2021-11-30

**Authors:** Ahmed Gowida, Ahmed Farid Ibrahim, Salaheldin Elkatatny, Abdulwahab Ali

**Affiliations:** College of Petroleum Engineering & Geosciences, King Fahd University of Petroleum and Minerals, Dhahran 31261, Saudi Arabia

## Abstract

The least principal stresses of downhole formations include minimum horizontal stress (*σ*_min_) and maximum horizontal stress (*σ*_max_). *σ*_min_ and *σ*_max_ are substantial parameters that significantly affect the design and optimization of the drilling process. These stresses can be estimated using theoretical equations in addition to some field tests, i.e., leak-off test to include the effect of tectonic stress. This approach is associated with many technical and financial issues. Therefore, the objective of this study is to provide a novel machine learning-based solution to estimate these stresses while drilling. First, new models were developed using artificial neural network (ANN) to directly predict *σ*_min_ and *σ*_max_ from the drilling data; which are injection rate (Q), standpipe pressure (SPP), weight on bit (WOB), torque (T), and rate of penetration (ROP). Such data are always available while drilling, and hence, no additional cost is required. Actual data from a Middle Eastern field were collected, statistically analyzed, and fed to the models. First, the models' predictions showed a significant match with the actual stress values with a correlation coefficient (R-value) exceeding 0.90 and a mean absolute average error (MAPE) of 0.75% as a maximum. Second, new empirical equations were generated based on the developed ANN-based models. The new equations were then validated using another unseen dataset from the same field. The predictions had an R-value of 0.98 and 0.93 in addition to MAPE of 0.36% and 0.96% for *σ*_min_ and *σ*_max_ models, respectively. The results demonstrated the outperformance of the developed ANN-based equations to estimate the least principal stresses from the drilling data with high accuracy in a timely and economically effective way.

## 1. Introduction

### 1.1. Background

The in situ stress state of earth's subterranean formations can be defined by three mutually orthogonal stress components. These principal stresses are the vertical stress (*σ*_*v*_) and the least principal stresses; the maximum horizontal stress (*σ*_max_) and the minimum horizontal stress (*σ*_min_). Based on the relative magnitude of the three principle stresses, the stress regime can be classified to normal faulting (*σv* > *σ*_max_ > *σ*_min_), strike-slip (*σ*_max>_*σ*v> *σ*_min_), and thrust faulting (*σ*v > *σ*_min_ > *σ*_max_) [1].

Estimation of these stresses is substantial for well planning since it defines the stress concentration around the wellbore. Therefore, it has a great impact on the optimization of the drilling process and maintaining the well integrity [2]. The availability of such information could help avoid many drilling-related issues such as stuck pipe and loss of circulation, by helping better design the safe drilling window, stable drilling trajectories, and set safe casing setting depths. [1].

The vertical stress (*σ*_v_) at a certain depth can be calculated using the densities of the overlying formations that could be obtained from the density log [3]. The minimum horizontal stress (*σ*_min_) can be directly measured by employing some field tests, i.e., leak-off test, minifrac test, and step-rate test, [1, 4, 5]. Unlike *σ*_min_, the maximum horizontal stress (*σ*_max_) is commonly estimated based on the values of *σ*_v_ and *σ*_min_, using some theoretical and empirical correlations [6, 7]. Since the field tests applied to measure *σ*_min_ are costly, time-consuming, and only applied at specific depths, different theoretical models have been developed, i.e., poroelastic strain models, to estimate the downhole stresses indirectly [1, 8–11]. Such models are based on the in situ measurements of some geomechanical parameters such as static elastic modulus, static Poisson's ratio, and elastic strains. These parameters are accurately measured in the lab of retrieved core samples that imitate the in situ conditions of the downhole formations [10]. To have a continuous profile of such geomechanical parameters, such lab measurements are correlated to the continuous logging data. Furthermore, at least one direct field test, i.e., leak-off test, should be conducted to calibrate these profiles and the effect of the tectonic stresses should be included so that they would effectively represent the in situ stress state of the downhole formations [12–14]. However, the well-logging process is commonly applied after drilling the wellbore to avoid the harsh drilling environment [15]. Thus, the logging data are not always accessible while drilling which would accordingly hinder the real-time estimation of the in situ stress state of the downhole formations. The availability of downhole stresses data during drilling is very crucial to optimize the drilling operation, reduce the nonproductive time (NPT), and prevent the collapse of downhole formations, so that the well integrity would be maintained.

During the drilling process, many sensors are installed to measure different parameters that reflect the performance of the drilling operation and the nature of the drilled formations. These parameters, known as the drilling parameters, include injection rate (Q), standpipe pressure (SPP), weight on bit (WOB), torque (T), and rate of penetration (ROP). Such data are always available while drilling and vary based on the properties of the drilled formations. The drilling parameters (Q, SPP, T, WOB, and ROP) practically reflect the drillability of the downhole formations. How easily the formations can be drilled is directly controlled by the stress concentration around the wellbore which is the key factor for the stability of the wellbore while drilling and maintaining its integrity [16]. The stress concentration around the wellbore is basically described by the hoop and radial stresses that are calculated based on the least principal stress values [10]. Practically, the two parameters, namely, WOB and Q, are controlled during the drilling operations. The initial values for these parameters are usually set based on the data available from offset wells and the experience of the drilling engineer with the area. Then, the set values of these parameters would be adjusted while drilling according to the drillability of the downhole formations which mainly depend on the stress concentration around the wellbore [17, 18]. Accordingly, this would be translated into the measured values of SPP, T, and ROP. For instance, the drillability of highly stressed formations such as shale would be different from normally stressed zones, and this would require adjusting the controlled drilling parameters accordingly. However, the shape of the downhole cuttings would be different, and in turn, the applied pumping rate (*Q*) would be adjusted to adapt such changes and achieve effective hole cleaning. Similarly, as the formation stress increases, it becomes difficult to drill, so higher WOB is required for effective rock crushing. Following this look, the drilling parameters, in practice, are usually adjusted according to the drillability of the formations.

Many studies have used such drilling parameters to estimate different mechanical properties of the downhole formations such as unconfined compressive strength, elastic moduli, and Poisson's ratio [19–22]. Recently, several machine learning (ML) techniques have been applied on a wide scale in the petroleum industry [23–26]. These applications aim at the best use of the big data available and support the fourth revolution for drilling automation and optimization.

Minimum horizontal stress (*σ*_min_) and the maximum horizontal stress (*σ*_max_) of downhole formations are essential for the design and optimization of the drilling process in addition to designing hydraulic fracturing operations. Theoretical equations can be used to estimate *σ*_min_ and *σ*_max_. These equations depend on some field tests, i.e., leak-off test to include the effect of tectonic stress. In addition, some in-situ geomechanical parameters can be estimated using retrieved core samples, and then the experimental results will be used to calibrate the logging data to have a continuous profile. Hence, this approach has many technical and financial issues. Therefore, the main objective of this study is to apply an ML approach i.e., artificial neural network (ANN) to predict the least principal stresses *σ*_min_ and *σ*_max_ using readily available drilling parameters. Then, state-of-the-art equations would be developed (a white-box model) to estimate the least principal stresses directly from the drilling data, based on the developed ML models. This would help provide a continuous profile of *σ*_min_ and *σ*_max_ directly while drilling without any additional costs in a timely and effective way.

### 1.2. Stresses Determination

In this study, the poroelastic model was used to determine the least principal stresses from (1) and (2) [9, 16].

(1) $$\begin{array}{c} \sigma_{\min}=\frac{PR_{s}}{1-PR_{s}}\sigma_{v}-\frac{PR_{s}}{1-PR_{s}}\alpha P_{f}+\alpha P_{f}+\frac{E_{s}}{1-PR_{s}^{2}}\varepsilon_{x}+\frac{PR_{s}\times E_{s}}{1-PR_{s}^{2}}\varepsilon_{y}, \end{array}$$

(2) $$\begin{array}{c} \sigma_{\max}=\frac{PR_{s}}{1-PR_{s}}\sigma_{v}-\frac{PR_{s}}{1-PR_{s}}\alpha P_{f}+\alpha P_{f}+\frac{E_{s}}{1-PR_{s}^{2}}\varepsilon_{y}+\frac{PR_{s}\times E_{s}}{1-PR_{s}^{2}}\varepsilon_{x}, \end{array}$$

where *PR*_*s*_ is the static Poisson's ratio; *σ*_v_ is the vertical (overburden) stress component; *α* is Biot's elastic coefficient; and *ε*_*x*_ and *ε*_*y*_ are the elastic strains in the *σ*_min_ and *σ*_max_ directions, respectively.

The overburden stress *σ*_v_ was firstly estimated using the formation bulk-density log (RHOB) along the depth of interest using the following equation:

(3) $$\begin{array}{c} \sigma_{v}=\int_{0}^{z}\rho \left(z\right)g\;dz, \end{array}$$

where *ρ*(*z*) is the formation density at a certain depth of *z* and *g* is the gravitational acceleration.

Secondly, the acoustic and RHOB logs were used to estimate the dynamic elastic modulus (*E*_*d*_) and dynamic Poisson's ratio (PR_*d*_). Since the wellbore failure is slow and the wave propagation in the layers is a high-frequency phenomenon, *E*_*d*_ was transformed to the static elastic modulus (*E*_*s*_) [27, 28]. Thus, *E*_s_ values were correlated with *E*_d_ using the lab measurements of the retrieved core samples from the wells.

The elastic strains *ε*_*x*_ and *ε*_*y*_ were initially considered equal in equation (1) to estimate initial values of *σ*_min_. The minimum horizontal stress was then calibrated using an in situ field test; leak-off test. The ratio (*ε*_*x*_/*ε*_*y*_) varied iteratively to achieve an acceptable match between the calculated and measured *σ*_min_ values. Finally, the *σ*_min_ and *σ*_max_ profiles were generated and used as the outputs for the proposed models.  Figure 1 shows the generated principal stress profiles for the area under study along the depth of interest. It is clear from Figure 1 that the stress regime in the presented case is normal faulting where *σv* > *σ*max > *σ*min.

## 2. Data Analysis and Processing

### 2.1. Data Description

Field data representing a complex carbonate reservoir were collected from two wells, Well A and Well B, in a Middle Eastern field. The data, 2187 data points, involve the drilling data and the corresponding in situ minimum and maximum horizontal stresses, *σ*_min_ and *σ*_max_. The drilling data comprise Q, SPP, WOB, T, and ROP. The data from Well A were used for building the models, while the data from Well B were used for the verification process of the developed models.

The statistical analysis listed in Table 1 shows different descriptive measures, i.e., range, mean, standard deviation (STD), and skewness. These measures gave descriptive insights about the data distribution and coverage. Having a wide data range with a representative distribution, as listed in Table 1, a substantial base is provided to develop a reliable model that could capture the nature of the problem with more confidence. The ranges of the data are as follows: Q, 191.54–289.92 gpm; SPP, 1748.58–3252.60 psi; T, 2.60–3.79 kft.lbf; WOB, 5.75–18.94 klb; ROP, 3.20–73.17 ft/hr; *σ*_min_, 11240.43–12361.17 psi; and *σ*_max_, 12308.02–14599.67 psi.  Figure 2 shows a graphical distribution of the drilling data used as inputs for the proposed model.

A specially designed Python code was developed to preprocess the data. First, the dataset was filtered from any missing data, duplicated information, negative values, and unreasonable values that violate the engineering sense. Then, the data outliers were removed using different approaches, i.e., moving mean and quartiles. The data preprocessing step is crucial for enhancing the quality of the data and in turn increases the potential to have an accurate predictive model [29].

The relative dependency of the output was then studied with each input parameter using Pearson's correlation coefficient (*R*-value). The R-value ranges from −1 to +1 in the way that the higher the R-value is, the stronger the linear relationship exists. Positive R-values indicate a direct relationship, while negative R-values indicate an inverse relationship between the input and the output parameters. R-values approaching zero show almost no linear relationship between the two parameters [30]. As shown in Figure 3, *σ*_min_ data have R-values of 0.65, 0.85, 0.59, 0.64, and −0.48 with Q, SPP, T, WOB, and ROP, respectively. Similarly, *σ*_max_ has relatively high positive *R*-values almost exceeding 0.50 with all the inputs except −0.34 with ROP. This indicates the noticeable dependence of both *σ*_min_ and *σ*_max_ on the selected input features. The uniqueness of the ML is that ML can be able to find the direct and the indirect relationships between the input and the output parameters. To the best of the author's knowledge, there is no direct relationship between the drilling parameters and the in situ stresses; however, as the formation stress increases, the drillability of the formation decreases [17]. [31–34] showed that rock cuttability decreased in the stressed formations. And that can be translated to lower ROP and higher T as the formation stress increases. Moreover, as the formation becomes difficult to be drill, higher WOB and horse power (Q^*∗*^SPP) is required to drill the formation, which is in agreement with the correlation coefficient result that is shown in Figure 3.

## 3. Model Development

The data collected from Well A were used for building the proposed ANN models to predict *σ*_min_ and *σ*_max_ as outputs based on the drilling data as inputs.

### 3.1. Artificial Neural Network (ANN)

ANN is a supervised-learning ML approach that is capable of dealing with highly complex problems. Based on the literature, ANN has been widely applied in many petroleum-related applications such as the predictions of the mechanical properties of the downhole formations based on the drilling parameters. Examples of these applications are the prediction of Poisson's ratio and unconfined compressive strength (UCS) [21, 35–38]. The typical structure of ANN architecture comprises three basic types of layers: input layer, hidden layer(s), and output layer. Building an ANN-based model involves processing the data through these layers starting from the input layer, then the neurons in the hidden layer(s), and eventually resulting in the target in the output layer [39]. The connections between the layers are typically controlled by a set of weights and biases that are updated iteratively during the optimization process to ultimately achieve the lowest possible loss in the objective function [40, 41].

### 3.2. Stresses Prediction Using ANN-Based Model

In this study, new ANN-based models were developed to estimate *σ*_min_ and *σ*_max_ based on the drilling data as inputs. A MATLAB code was developed to randomly divide the selected dataset into two groups: 80% of the data for training and 20% testing. The training set was used to train the model to optimize its hyperparameters. During the optimization process, the results of the models were internally tested to evaluate the selected hyperparameters. For each trial, the predictions were evaluated using the R-value and the mean absolute percentage error (MAPE) between the actual and predicted output values for the training and testing processes. The objective of this step is to identify the hyperparameters that could achieve the lowest possible prediction error through many iterative trials. Afterwards, the model with the optimized hyperparameters was evaluated using the testing set to estimate the generalization error of the optimized model [42]. Different options of the ANN parameters were tested to optimize the network. These parameters are the number of hidden layers, number of neurons in each hidden layer, training algorithms, transfer functions, and the learning rate.  Table 2 lists the tested options of the network parameters for optimizing the developed ANN-based models.  Figure 4 summarizes the workflow adopted while developing the ANN models.

## 4. Results and Discussion

### 4.1. *σ*_min_ Prediction Model

The developed model was trained using the Levenberg–Marquardt algorithm (trainlm) to tune the ANN parameters. Different hyperparameters were tested to optimize the architecture of the ANN-based model. Different numbers of hidden layers were tested between single to four layers, and the optimized number was selected to be a single layer. The number of neurons was selected to be 15 neurons after testing the number of the neurons between 5 and 40 neurons. Different training to testing splitting ratios from 60/40 to 90/10 were tested. The best model performance was found with an 80/20 splitting ratio. The optimized training algorithm and transfer function were found to be trainlm and Log-sigmoidal transfer function (logsig) for the input layer, respectively. The learning rate of the ANN model was selected to be 0.12.

Figure 5 shows a typical architecture of the developed ANN-based model. A significant match was found between the predicted and actual *σ*_min_ as shown in Figure 6, confirmed by the R-value of 0.98 and 0.97 MAPE not exceeding 0.36% both for the training and testing processes, respectively.

### 4.2. *σ*_max_ Prediction Model

Similarly, another model was developed using ANN to predict *σ*_max_ based on the drilling parameters. The optimization process of the *σ*_max_ model yielded a network structure of a single hidden layer with 35 neurons. A tan-sigmoidal transfer function was used for the input layer, while a linear function was selected for the output layer using the “trainlm” algorithm for training the model. The predictions of the developed model showed a narrow scatter around the 45 lines of the crossplots between the actual and the predicted *σ*_max_ values as shown in Figure 7. This indicates the high accuracy of the model predictions that is confirmed by the low MAPE of 0.74%, and 0.75% for the training and testing processes, respectively. Besides, the high R-value exceeds 0.90 for both. The summary of the prediction evaluation of the developed models is listed in Table 3, in terms of R-value, MAPE, and root-mean squared error (RMSE) for both the training and testing processes.

## 5. Empirical Equations for Estimating *σ*_min_ and *σ*_max_

This study aims at introducing ML-based models to predict *σ*_min_ and *σ*_max_ in a white-box model to demulsify the black-box nature of the ML models. Therefore, the weights and biases of the optimized models were extracted to imitate the workflow of the developed ANN models. Accordingly, new equations, equations (4) and (5), were developed to estimate *σ*_min_ and *σ*_max_, respectively:

(4) $$\begin{array}{c} \sigma_{\min}=560.37\times {\left(\sigma_{\min}\right)}_{\text{normalized}}+11800.80, \end{array}$$

(5) $$\begin{array}{c} \sigma_{\max}=1145.83\times {\left(\sigma_{\max}\right)}_{\text{normalized}}+13453.84, \end{array}$$

where (*σ*_min_)_normalized_ and (*σ*_max_)_normalized_ are the normalized forms of *σ*_min and_*σ*_max_, respectively.

As a first procedure to use the ANN-based equations, the input parameters should be initially normalized using the following equation:

(6) $$\begin{array}{c} X_{\text{normalized}}=2\times \left(\frac{X-X_{\min}}{X_{\max}-X_{\min}}\right)-1, \end{array}$$

where *X* is the actual value of the input parameter, *X*_min_ and *X*_max_ are the minimum and maximum values of the input parameter, respectively, and X_normalized_ is the normalized form of the input parameter. The minimum and maximum values of each parameter are listed in Table 1. Equations (7) and (8) are used to calculate the normalized forms of *σ*_min_ and *σ*_max_ to substitute (*σ*_min_)_normalized_ and (*σ*_max_)_normalized_ in Equation (4) and (5):

(7) $$\begin{array}{c} {\left(\sigma_{\min}\right)}_{\text{normalized}}=\left[\sum_{i=1}^{k}w_{2,i}\left(\frac{1}{1+e^{-\left(\left(w_{1_{i,1}}\times Q_{n}\right)+\left(w_{1_{i,2}}\times SPP_{n}\right)+\left(w_{1_{i,3}}\times WOB_{n}\right)+\left(w_{1_{i,4}}\times T_{n}\right)+\left(w_{1_{i,5}}\times ROP_{n}\right)+b_{1,i}\right)}}\right)\right]+b_{2}, \end{array}$$

(8) $$\begin{array}{c} {\left(\sigma_{\max}\right)}_{\text{normalized}}=\left[\sum_{i=1}^{k}w_{2,i}\left(\frac{2}{1+e^{-2\left(\left(w_{1_{i,1}}\times Q_{n}\right)+\left(w_{1_{i,2}}\times SPP_{n}\right)+\left(w_{1_{i,3}}\times WOB_{n}\right)+\left(w_{1_{i,4}}\times T_{n}\right)+\left(w_{1_{i,5}}\times ROP_{n}\right)+b_{1,i}\right)}}-1\right)\right]+b_{2}, \end{array}$$

where *k* is the total number of neurons in the hidden layer; *w*_2_is the vector of the optimized weights between the hidden layer and the output layer; *w*_1_ is the matrix of the optimized weights between the hidden layer and the input layer; *b*_1_ is the vector of the optimized biases between the hidden layer and the input layer; and *b*_2_ is the optimized bias between the hidden layer and the output layer. *Q*_n_, SPP_n_, WOB_n_, *T*_n_, and ROP_n_ are the normalized forms of the input parameters and can be calculated using Equation (6). The optimized weights and biases extracted from the developed ANN-based *σ*_min_ and *σ*_max_ models are listed in Tables 4 and 5, respectively. This is to substitute the weights and biases in Equations (7) and (8). The input parameters should be measured in the following units: Q in gpm, SPP in psi, WOB in klb, T in klb.ft, and ROP in ft/hr.

## 6. Model Verification

To verify the performance of the novel ANN-based equations, the dataset from Well B (386 data points) was used to validate the developed equations. The data involved the drilling data (Q, SPP, WOB, T, and ROP) and *σ*_min_ and *σ*_max_ at the corresponding depths. The drilling data were used as inputs for the developed equations. Then the results were compared with the actual *σ*_min_ and *σ*_max_ values. A remarkable match was noticed between the predicted and the actual *σ*_min_ and *σ*_max_ values as shown in Figure 8. The R-value was 0.98 and 0.93 for *σ*_min_ and *σ*_max_ predictions, respectively. The MAPE did not exceed 0.96% for both. These results revealed the outperforming accuracy of the developed ANN-based equations to estimate *σ*_min_ and *σ*_max_ from the drilling data and provided the capability of generating a real-time stress profile for the downhole formations while drilling.

It should be highlighted that the application of the developed equations is recommended only for carbonate formations because different responses in the drilling data, mechanical properties, and stress concentrations may be encountered for other types of formations. Furthermore, it is recommended to have the inputs within the same range and units listed in Table 1 to ensure reliable results.

## 7. Conclusions

In this study, new ML-based models were developed using ANN to predict *σ*_min_ and *σ*_max_ of the downhole formations using the readily available drilling data, namely, Q, SPP, T, WOB, and ROP, as inputs. The outcomes of this study are summarized as follows:

- The developed ANN-based models predicted the stress values with accuracy exceeding 90% and mean absolute percentage error (MAPE) of 0.75% compared to the actual values.
- Novel equations were extracted from the developed ANN-based models to estimate *σ*_min_ and *σ*_max_ using the optimized weights and biases of the ANN models.
- The extracted ANN-based equations were validated using unseen data from the same field, where the MAPE did not exceed 0.96%.

The results demonstrated the robustness of the ANN model to predict *σ*_min_ and *σ*_max_ from the drilling data to provide continuous profiles of these stresses while drilling and in turn help avoid many wellbore-instability issues in addition to maintaining the well integrity.

The current study uses the drilling parameters to predict the maximum and minimum horizontal stresses. The drilling data were collected from real-time sensors after optimizing the controllable drilling parameters such as WOB, RFP, and flow rate.

## Figures and Tables

**Figure 1:** Principal stress profile for the area under study.

**Figure 2:** Graphical presentation for the drilling data used for building the ANN models.

**Figure 3:** A graphical presentation of the correlation coefficient R-value between *σ*_min_ and *σ*_max_ with input data (drilling data).

**Figure 4:** A flowchart for the workflow followed while developing the ANN-based models.

**Figure 5:** A typical architecture of the developed ANN-based models.

**Figure 6:** Crossplots between the actual and predicted *σ*_min_ using the developed ANN-based model for (a) training and (b) testing processes.

**Figure 7:** Crossplots between the actual and predicted *σ*_max_ for the developed ANN-based model for (a) training and (b) testing processes.

**Figure 8:** Prediction performance of the developed ANN-based equations (actual vs. predicted stresses) for the verification process: (a) *σ*_min_ prediction (b) *σ*_max_ prediction.

**Table 1:** Descriptive statistical analysis of the dataset used in this study.

Parameter	*Q* (gpm)	SPP(psi)	T (kft.lbf)	WOB (klb)	ROP (ft/hr)	*σ*_min_ (psi)	*σ*_mzx_ (psi)
Minimum	191.54	1748.58	2.60	5.75	3.20	11240.43	12308.02
Maximum	289.92	3252.60	3.79	18.94	73.17	12361.17	14599.67
Range	98.38	1504.02	1.19	13.19	69.97	1120.74	2291.65
Mean	242.15	2759.52	3.07	10.31	22.27	11855.70	13731.48
STD	20.12	342.65	0.26	3.10	12.02	302.36	487.08
Skewness	−1.31	−1.12	0.95	0.76	1.05	−0.15	−0.42

**Table 2:** Summary of the optimization process of the developed ANN-based model.

Parameter	Optimized parameters	
	*σ*_min_ model	*σ*_max_ model
Number of hidden layers	Single hidden layer	
Number of neurons in each layer	15	35
Split ratio	(Training/testing) 0.8/0.2	
Training algorithms	Trainlm	
Transfer function	Logsig	Tansig
Learning rate	0.12	

**Table 3:** Summary of the performance of the developed ANN-based models.

Model	Training Process			Testing Process		
	*R*-value	MAPE (%)	RMSE	*R*-value	MAPE (%)	RMSE
*σ*_min_	0.98	0.36	60.37	0.97	0.29	48.57
*σ*_max_	0.96	0.74	136.25	0.96	0.75	129.51

**Table 4:** The optimized weights and biases of the developed ANN-based model to predict *σ*_min_.

*I*	*W*_1_*i*,*j*__						*W*_2_*i*__	*b*_1,i_	*b*_2_
	*j* = 1		*j* = 2	*j* = 3	*j* = 4	*j* = 5			
1	0.653		−2.017	6.168	−6.467	2.957	−0.363	0.379	0.481
2	−3.731		7.783	−0.918	−0.988	0.579	−2.357	−2.552	
3	11.880		9.908	1.902	1.074	−4.115	−3.858	−5.135	
4	−0.956		7.366	−0.953	0.713	3.276	1.281	−1.135	
5	4.816		8.946	−2.218	0.170	1.409	−3.243	−2.571	
6	−4.431		−1.371	−1.022	−2.537	0.786	−2.683	−0.397	
7	−0.339		0.733	1.250	3.444	1.301	1.464	−1.011	
8	1.520		0.881	−1.025	1.345	−0.458	−6.470	−0.439	
9	13.907		11.934	1.574	0.449	−4.262	4.254	−6.812	
10	1.046		8.303	−3.238	−0.367	0.403	5.115	−2.807	
11	2.097		2.800	−1.399	0.553	−0.719	4.314	−3.129	
12	−1.530		−0.759	−2.516	1.398	0.005	−1.618	0.148	
13	3.257		−0.022	1.328	−0.005	−0.315	−6.300	−1.223	
14	3.930		−5.095	3.617	0.298	−1.285	2.611	0.732	
15	1.121		4.980	−3.389	0.046	0.650	3.910	4.241	

**Table 5:** The optimized weights and biases of the developed ANN-based model to predict *σ*_max_.

*I*	*W*_1_*i*,*j*__					*W*_2_*i*__	*b*_1,i_	*b*_2_
	*j* = 1	*j* = 2	*j* = 3	*j* = 4	*j* = 5			
1	−5.288	0.974	0.115	−0.124	0.237	2.121	−0.633	1.772
2	−0.020	3.497	2.157	0.157	2.459	−0.857	1.606	
3	−4.615	−0.558	−0.743	0.988	−0.925	−1.908	−0.092	
4	−2.858	−0.075	−2.373	0.783	−1.055	−1.383	−0.509	
5	−1.201	−1.491	−0.970	−0.522	−0.885	3.055	−0.035	
6	−0.756	1.804	4.202	1.636	−1.023	1.835	3.599	
7	−0.002	−1.251	−4.740	2.218	−0.499	1.323	−1.971	
8	−4.088	1.246	2.770	−0.589	0.330	−2.059	1.539	
9	2.196	1.176	−1.558	−2.904	−2.890	0.659	1.519	
10	0.519	1.456	−1.624	1.092	−0.417	−2.393	0.747	
11	−3.117	−2.333	−1.600	−0.911	−0.393	−1.537	0.218	
12	−0.026	0.495	2.698	1.203	−0.665	−3.343	2.087	
13	−3.189	0.415	0.263	3.192	−0.008	−1.378	1.887	
14	−2.627	1.138	−0.152	−0.991	0.599	−2.080	0.345	
15	−0.748	0.988	−0.362	2.850	−1.012	1.309	1.783	
16	−1.820	−0.330	5.310	−0.836	2.682	1.322	2.900	
17	4.885	−0.756	−0.698	−4.450	1.975	−0.703	−1.525	
18	1.690	4.334	−2.065	2.208	−0.449	2.556	0.216	
19	2.966	0.747	1.833	−1.345	−0.235	1.933	−2.519	
20	0.710	1.635	0.142	0.234	2.167	1.664	0.974	
21	−0.775	1.511	2.444	−1.423	0.499	2.918	1.118	
22	−1.433	1.751	−0.098	2.574	0.924	1.049	0.727	
23	−0.376	1.619	1.941	−1.190	−2.214	−0.530	0.037	
24	0.571	−0.637	−1.583	1.343	0.394	−2.217	1.060	
25	5.831	0.459	−0.280	0.811	−0.423	−2.284	−2.314	
26	3.484	−3.748	3.357	−5.355	1.395	−0.355	0.712	
27	−2.568	−1.966	0.084	−0.359	−1.958	2.117	−0.860	
22	1.083	0.485	−4.025	0.816	−1.657	2.744	−2.142	
29	−2.825	0.173	4.042	−0.750	0.857	2.337	2.254	
30	−0.017	−1.234	−4.583	−1.940	0.968	−1.241	−2.621	
31	1.081	−0.800	0.352	−1.558	0.610	−3.118	1.441	
32	−2.956	1.570	0.844	−0.173	0.263	−2.507	−1.213	
33	0.958	−0.203	1.742	−1.198	−1.032	−2.362	−1.351	
34	2.337	6.044	−1.494	1.849	−0.748	−1.676	−0.694	
35	1.236	0.410	−0.855	−2.636	−0.213	0.856	0.355	

## Data Availability

The manuscript contains most of the data, and a detailed sample will be provided upon request.

## Abbreviations

*σ*_min_: Minimum horizontal stress
*σ*_max_: Maximum horizontal stress
ANN: Artificial neural network
Q: Mud injection rate
SPP: Standpipe pressure
T: Torque
WOB: Weight on bit
R: Correlation coefficient
ROP: Rate of penetration
gpm: Gallon per minute
MAPE: Mean absolute average error
RMSE: Root-mean-squared error
trainlm: Levenberg–Marquardt
tansig: Hyperbolic tangent sigmoid transfer function
logsig: Log-sigmoid transfer function
NPT: Nonproductive time
STD: Standard deviation
PR_s_: Static Poisson's ratio
UCS: Unconfined compressive strength
*σ*_v_: Vertical (overburden) stress component
*α*: Biot's elastic coefficient
*ε*_*x*_ and *ε*_*y*_: Elastic strains in the *σ*_min_ and *σ*_max_ directions, respectively.

## References

[1] Zoback M. D., Barton C. A., Brudy M. (2003). Determination of stress orientation and magnitude in deep wells. *International Journal of Rock Mechanics and Mining Sciences*.

[2] Al-Zankawi O., Belhouchet M., Abdessalem A. Real-time integration of geo-mechanics to overcome drilling challenges and low NPT.

[3] McGarr A., Gay N. C. (1978). State of stress in the Earth’s crust. *Annual Review of Earth and Planetary Sciences*.

[4] Carnegie A., Thomas M., Efnik M. S., Hamawi M., Akbar M., Burton M. An advanced method of determining insitu reservoir stresses: wireline conveyed micro-fracturing.

[5] Nolte K. G. (1988). *Principles for Fracture Design Based on Pressure Analysis*.

[6] Binh N. T. T., Tokunaga T., Goulty N. R., Son H. P., Van Binh M. (2011). Stress state in the cuu long and nam con son basins, offshore vietnam. *Marine and Petroleum Geology*.

[7] Zang A., Stephansson O., Heidbach O., Janouschkowetz S. (2012). World stress map database as a resource for rock mechanics and rock engineering. *Geotechnical & Geological Engineering*.

[8] Anderson E. M. (1905). The dynamics of faulting. *Transactions of the Edinburgh Geological Society*.

[9] Blanton T. L., Olson J. E. (1999). Stress magnitudes from logs: effects of tectonic strains and temperature. *SPE Reservoir Evaluation and Engineering*.

[10] Fjar E., Holt R. M., Raaen A. M., Horsrud P. (2008). *Petroleum Related Rock Mechanics*.

[11] Terzaghi K. (1925). *Erdbaumechanik auf bodenphysikalischer Grundlage*.

[12] Fan X., Gong M., Zhang Q., Wang J., Bai L., Chen Y. (2014). Prediction of the horizontal stress of the tight sandstone formation in eastern Sulige of China. *Journal of Petroleum Science and Engineering*.

[13] Meng Z., Zhang J., Wang R. (2011). In-situ stress, pore pressure and stress-dependent permeability in the Southern Qinshui Basin. *International Journal of Rock Mechanics and Mining Sciences*.

[14] Rasouli V., Pallikathekathil Z. J., Mawuli E. (2011). The influence of perturbed stresses near faults on drilling strategy: a case study in Blacktip field, North Australia. *Journal of Petroleum Science and Engineering*.

[15] Jackson C. E., Heysse D. R. Improving fonnation evaluation by resolving differences between lwd and wireline log data.

[16] Abdideh M., Fathabadi M. R. (2013). Analysis of stress field and determination of safe mud window in borehole drilling (case study: SW Iran). *Journal of Petroleum Exploration and Production Technology*.

[17] Prasad B. S., Murthy V., Pandey S. K. Investigations on rock drillability applied to underground mine development vis-à-vis drill selection.

[18] Hui L., Rui G., Junchang D., Li L., Yang L., Yingjie Y. (2013). Productivity evaluation and influential factor analysis for Sarvak reservoir in South Azadegan oil field, Iran. *Petroleum Exploration and Development*.

[19] Asadi A. (2017). Application of artificial neural networks in prediction of uniaxial compressive strength of rocks using well logs and drilling data. *Procedia Engineering*.

[20] Gowida A., Elkatatny S., Moussa T. Comparative analysis between different artificial based models for predicting static Poisson’s ratio of sandstone formations.

[21] He M., Zhang Z., Ren J. (2019). Deep convolutional neural network for fast determination of the rock strength parameters using drilling data. *International Journal of Rock Mechanics and Mining Sciences*.

[22] Siddig O. M., Al-Afnan S. F., Elkatatny S. M., Abdulraheem A. (2021). Drilling data-based approach to build a continuous static elastic moduli profile utilizing artificial intelligence techniques. *Journal of Energy Resources Technology*.

[23] Ashrafi S. B., Anemangely M., Sabah M., Ameri M. J. (2019). Application of hybrid artificial neural networks for predicting rate of penetration (ROP): a case study from Marun oil field. *Journal of Petroleum Science and Engineering*.

[24] Mehrad M., Bajolvand M., Ramezanzadeh A., Neycharan J. G. (2020). Developing a new rigorous drilling rate prediction model using a machine learning technique. *Journal of Petroleum Science and Engineering*.

[25] Otchere D. A., Arbi Ganat T. O., Gholami R., Ridha S. (2021). Application of supervised machine learning paradigms in the prediction of petroleum reservoir properties: comparative analysis of ANN and SVM models. *Journal of Petroleum Science and Engineering*.

[26] Qing W., Bangert P. (2021). Chapter 9-global practice of AI and big data in oil and gas industry. *Machine Learning and Data Science in the Oil and Gas Industry*.

[27] Afsari M., Ghafoori M., Roostaeian M., Haghshenas A., Ataei A., Masoudi R. Mechanical earth model (MEM): an effective tool for borehole stability analysis and managed pressure drilling (case study).

[28] Keshavarzi R., Jalili S. (2014). Building a mechanical earth model and its application in a geomechanical analysis of hydraulic fracture behaviour in naturally fractured reservoirs. *European Journal of Environmental and Civil Engineering*.

[29] Kotsiantis S. B. (2012). Use of machine learning techniques for educational proposes: a decision support system for forecasting students’ grades. *Artificial Intelligence Review*.

[30] Sedgwick P. (2012). Pearson’s correlation coefficient. *BMJ*.

[31] Gehring K. (1995). Design criteria for TBM’s with respect to real rock pressure. *Proceedings of the Tunnel Boring Machines: Trends in Design and Construction of Mechanized Tunnelling*.

[32] Innaurato N., Oggeri C., Oreste P., Vinai R. (2007). Experimental and numerical studies on rock breaking with TBM tools under high stress confinement. *Rock Mechanics and Rock Engineering*.

[33] Innaurato N., Oreste P. (2011). Theoretical study on the TBM tool-rock interaction. *Geotechnical & Geological Engineering*.

[34] Li X., Wang S. (2018). Experimental investigation of the influence of confining stress on hard rock fragmentation using a conical pick. *Rock Mechanics and Rock Engineering*.

[35] Ahmed A., Elkatatny S., Abdulraheem A. (2021). Real-time static Poisson’s ratio prediction of vertical complex lithology from drilling parameters using artificial intelligence models. *Arabian Journal of Geosciences*.

[36] Elkatatny S. (2021). Real-time prediction of the dynamic young’s modulus from the drilling parameters using the artificial neural networks. *Arabian Journal for Science and Engineering*.

[37] Gowida A., Elkatatny S., Gamal H. (2021). Unconfined compressive strength (UCS) prediction in real-time while drilling using artificial intelligence tools. *Neural Computing & Applications*.

[38] Jamshidi E., Arabjamaloei R., Hashemi A., Ekramzadeh M. A., Amani M. (2013). Real-time estimation of elastic properties of formation rocks based on drilling data by using an artificial neural network. *Energy Sources, Part A: Recovery, Utilization, and Environmental Effects*.

[39] Lippmann R. (1987). An introduction to computing with neural nets. *IEEE ASSP Magazine*.

[40] Hinton G. E., Osindero S., Teh Y.-W. (2006). A fast learning algorithm for deep belief nets. *Neural Computation*.

[41] Nakamoto P. (2017). *Neural Networks & Deep Learning*.

[42] Xu Y., Goodacre R. (2018). On splitting training and validation set: a comparative study of cross-validation, bootstrap and systematic sampling for estimating the generalization performance of supervised learning. *Journal of Analysis and Testing*.

